The article "Somatostatin plus Ulinastatin in the Treatment of Severe Acute Pancreatitis and Its Effect on Serum Cytokine Levels" was retracted in 2023. Reasons: unreliable results or conclusions; concerns about the data; concerns about the peer review; concerns about the citations.

# Somatostatin plus Ulinastatin in the Treatment of Severe Acute Pancreatitis and Its Effect on Serum Cytokine Levels

**DOI:** 10.1155/2022/7223632

**Published:** 2022-06-09

**Authors:** Li Yang, Zhibin Zhao

**Affiliations:** Department of Gastroenterology, Taizhou People's Hospital, Taizhou 225300, China

## Abstract

**Objective:**

To investigate the effect of somatostatin combined with ulinastatin in the treatment of patients with severe acute pancreatitis and its effect on serum cytokine levels.

**Methods:**

This study is a retrospective trial. One hundred patients with severe acute pancreatitis in our hospital between March 2020 and May 2021 were recruited and assigned into the control group (ulinastatin alone) and experimental group (somatostatin plus ulinastatin) according to different treatment methods, 50 cases each. The clinical efficacy and serum cytokine levels of the two groups were compared.

**Results:**

Somatostatin plus ulinastatin was associated with a higher total effective rate versus ulinastatin alone (*p* < 0.05). After treatment, the experimental group observed significantly better interleukin-10 (IL-10), interleukin-18 (IL-18), and tumor necrosis factor-*α* (TNF-*α*) when compared with those in the control group (*p* < 0.05); somatostatin plus ulinastatin resulted in better serum amylase, blood calcium, blood urea nitrogen, blood sugar, and white blood cell count versus ulinastatin alone (*p* < 0.05).

**Conclusion:**

Somatostatin plus ulinastatin is a viable alternative in the treatment of patients with severe acute pancreatitis, with a remarkable efficacy profile. It is worthy of clinical application.

## 1. Introduction

Severe acute pancreatitis is a critical illness in pancreatitis characterized by sudden onset and critical conditions. Inappropriate treatment aggravates the condition and is accountable for over 25% acute pancreatitis-associated mortality [1, 2]. Clinically, surgery is the mainstay, yet strong evidence suggest that surgical treatment is associated with multiple complications, postoperative body pain, and slow postoperative recovery [3]. Fang et al. [4] proposed that drugs for conservative treatment might be a viable potion for patients with acute pancreatitis who are unwilling to undergo surgery. Somatostatin is one of the commonly used drugs in the clinical treatment of patients with pancreatitis by inhibiting the secretion of insulin and glucagon, thereby reducing the secretion of pancreas and gallbladder and contributing to gastrointestinal absorption and nutritional function [5, 6]. Ulinastatin, a class of broad-spectrum pancreatic enzyme inhibitors, inhibits the hydrolysis of amylase, lipase, trypsin, and lysozyme and is conducive to inhibit the secretion of trypsin and other pancreatic enzymes, thereby reducing the occurrence of inflammatory response and preventing the damage caused by self-digestion of the pancreas to tissues and organs [7]. However, few studies have been conducted on the efficacy of combination of the two drugs [8]. To fill the gap, this study analyzes the effect of somatostatin plus ulinastatin in the treatment of patients with severe acute pancreatitis and its impact on serum cytokine levels.

The article "Somatostatin plus Ulinastatin in the Treatment of Severe Acute Pancreatitis and Its Effect on Serum Cytokine Levels" was retracted in 2023. Reasons: unreliable results or conclusions; concerns about the data; concerns about the peer review; concerns about the citations.

## 2. Materials and Methods

### 2.1. Baseline Information

This study is a retrospective trial. One hundred patients with severe acute pancreatitis in Taizhou People's Hospital between March 2020 and May 2021 were recruited and assigned into the control group (ulinastatin alone) and experimental group (somatostatin plus ulinastatin) according to different treatment methods, 50 cases each. There were 27 males and 23 females in the control group, aged 35–65 years, with an average age of (48.61 ± 4.51) years. The experimental group included 25 males and 25 females, aged 36–63 years, with an average age of (48.50 ± 4.48) years. The baseline data in the two groups were balanced with good comparability. This study was reviewed and approved by the Taizhou People's Hospital, no. #17201.

### 2.2. Inclusion and Exclusion Criteria

Inclusion criteria: were as follows: severe acute pancreatitis was diagnosed by the laboratory blood test and abdominal color Doppler ultrasonography and the patients and their families were informed about the study and signed the informed consent. Exclusion criteria were as follows: patients with contradictions to somatostatin and ulinastatin and patients with poor compliance and communication disorder.

### 2.3. Treatment

The patients in the control group were treated with ulinastatin (Guangdong Tianpu Biochemical Pharmaceutical Co., Ltd., H19990132, 1 ml: 50000 U), 50000 U was added to 500 ml of 5% glucose injection for intravenous drip, once a day. On the basis of treatment in the control group, the patients in the experimental group were treated with somatostatin (Stilamin) (Serono, Switzerland, H20090929, powder injection 250 *μ*g), and 250 *μ*g was added to 500 ml of normal saline injection for intravenous drip, 2 times a day. The patients in both groups were treated for consecutive 7 days.

On the basis of Western medicine symptomatic treatment, traditional Chinese medicine treatment was supplemented. If the symptoms are red tongue, yellow and greasy coating, slippery pulse, and the syndrome of accumulation of dampness and heat, Dachaihu decoction was given to clear heat and dehumidify, clear the inside, and detoxify. Components of Dachaihu are as follows: *Bupleurum* 15 g, *Scutellaria baicalensis* 15 g, *Pinellia* 15 g, *Gardenia* 15 g, *Gentiana* 12 g, dandelion 15 g, raw rhubarb 10 g, Glauber's salt 20 g, *Magnolia* 15 g, and *Citrus aurantium* 15 g. If the tongue is red, the coating is thin and yellow, the pulse is stringy, and the syndrome is identified as liver stagnation and qi stagnation, Dachengqi decoction was given to sooth the liver and regulate qi, clear away heat and detoxify, and clear the body. Components of Dachengqi are as follows: *Bupleurum* 15 g, *Scutellaria baicalensis* 15 g, *Coptis chinensis* 12 g, costus root 12 g, corydalis tuber 15 g, betel nut 12 g, *Magnolia officinalis* 15 g, *Citrus aurantium* 15 g, raw rhubarb 10 g, and Glauber's salt 20 g. Both groups of patients were orally given Dachaihu decoction or Dachengqi decoction once a day according to the actual symptoms of the patients.

The article "Somatostatin plus Ulinastatin in the Treatment of Severe Acute Pancreatitis and Its Effect on Serum Cytokine Levels" was retracted in 2023. Reasons: unreliable results or conclusions; concerns about the data; concerns about the peer review; concerns about the citations.

### 2.4. Outcomes

(1) Clinical efficacy: cured: the patient's clinical symptoms disappeared and serum cytokine levels returned to normal; effective: the patient's clinical symptoms were significantly mitigated, and serum cytokine levels were close to those of mild patients; ineffective: the patient's clinical symptoms showed no improvement, and serum cytokine levels did not change significantly. Total effective rate = (number of cured cases + number of effective cases)/total number of cases × 100%. (2) Detection of serum cytokine levels: 10 ml of venous peripheral blood was collected from all patients before and after treatment, and blood was evenly divided into 2 samples. One blood sample was centrifuged, and the upper serum was taken to detect the levels of interleukin-10 (IL-10), interleukin-18 (IL-18), and tumor necrosis factor-*α* (TNF-*α*), and upper serum of the other blood samples was centrifuged to detect serum amylase, blood calcium, blood urea nitrogen, blood sugar, and white blood cell count.

### 2.5. Statistical Analysis

All data analyses were performed with the SPSS 21.0 software. Measurement data are described by mean ± standard deviation (*x* ± *s*) and were analyzed by the *t*-test; count data are expressed as number of cases (rate) and were verified via the *X*^2^ test. The level of significance was set at *p* < 0.05.

## 3. Results

### 3.1. Clinical Efficacy

Somatostatin plus ulinastatin was associated with a higher total effective rate versus ulinastatin alone (*p* < 0.05, Table 1).

### 3.2. IL-10, IL-18, and TNF-*α*

Before treatment, there was no significant difference in the levels of IL-10, IL-18, and TNF-*α* between the two groups (*p* > 0.05); after treatment, the experimental group observed significantly better IL-10, IL-18, and TNF-*α* when compared with those in the control group (*p* < 0.05, Table 2).

The article "Somatostatin plus Ulinastatin in the Treatment of Severe Acute Pancreatitis and Its Effect on Serum Cytokine Levels" was retracted in 2023. Reasons: unreliable results or conclusions; concerns about the data; concerns about the peer review; concerns about the citations.

### 3.3. Serum Amylase, Blood Calcium, Blood Urea Nitrogen, Blood Sugar, and White Blood Cell Count

Before treatment, the serum amylase, blood calcium, blood urea nitrogen, blood glucose, and white blood cell count in the two groups did not differ (*p* > 0.05); somatostatin plus ulinastatin resulted in better serum amylase, blood calcium, blood urea nitrogen, blood sugar, and white blood cell count versus ulinastatin alone (*p* < 0.05).

## 4. Discussion

Severe acute pancreatitis is clinically characterized by acute onset and rapid disease progression, threatening safety of the patient [9]. A wealth of evidence suggest that severe acute pancreatitis is associated with abnormal secretion of pancreatic juice and severe inflammatory response [10]. Overwhelming release of inflammatory factors leads to the increased permeability of the digestive tract, thereby aggravating the hemorrhage or necrosis of the pancreas and then inducing a chain reaction of organ failure [11]. Therefore, inhibiting the release of inflammatory factors in patients with severe acute pancreatitis has become the top priority of treatment [12].

Stilamin, one of the commonly used growth hormone-releasing inhibitory hormones in clinical practice, is predominantly used for the treatment of upper gastrointestinal bleeding and acute pancreatitis caused by gastric ulcers and displays an immunomodulatory effect [13]. It inhibits the secretion of growth hormone, insulin, and pepsin, as well as the endocrine secretion of the patient's pancreatic glands, thereby reducing the pancreatic enzyme activity of the patient's body [14]. Feng et al. found that Stilamin is capable to reducing the blood flow and pressure of the portal vein in patients and further slowing splanchnic blood flow [15]. Ulinastatin, a class of broad-spectrum pancreatic enzyme inhibitors, can effectively reduce the activity of trypsin, plasmin, and other pancreatic enzymes in patients, thereby inhibiting the occurrence of inflammatory reactions [16] and enhancing the immunity of body. Additionally, ulinastatin plays a pivotal role in reducing the release of lysosomal enzymes to ensure a stability of the lysosomal membrane [17]. In this study, we found that somatostatin plus ulinastatin was associated with a higher total effective rate versus ulinastatin alone [18]. Inflammatory factors that play a key role in the occurrence and development of severe acute pancreatitis mainly include IL-10, IL-18, and TNF-*α*. IL-10 can not only inhibit Th1 cell response and synthesis of cytokines but also suppress the antigen-presenting function and synthesis of cytokines of macrophages, which effectively promotes the proliferation, differentiation, and antibody production of B cells in patients. IL-18 can stimulate the cytotoxic activity of NK cells and lymphocytes in patients. Wang et al. found that the level of IL-18 is associated with the severity of acute pancreatitis. Therefore, the level of IL-18 serves as a major indicator to determine the severity of acute pancreatitis. The TNF-*α* is derived from the phagocytic cells, and overexpression of TNF-*α* leads to pancreatic tissue damage [19].

The article "Somatostatin plus Ulinastatin in the Treatment of Severe Acute Pancreatitis and Its Effect on Serum Cytokine Levels" was retracted in 2023. Reasons: unreliable results or conclusions; concerns about the data; concerns about the peer review; concerns about the citations.

In the present study, somatostatin plus ulinastatin resulted in superior IL-10, IL-18, and TNF-*α* versus ulinastatin alone. This would suggest a promising effectiveness profile of somatostatin plus ulinastatin in mitigating the inflammatory response in severe acute pancreatitis [20]. In keeping with our results, Li et al. [21] found that serum amylase, blood calcium, blood urea nitrogen, blood sugar, and white blood cell counts well reflect the pancreatic function and inflammatory response in patients with severe acute pancreatitis. Here, we observed that somatostatin plus ulinastatin resulted in better serum amylase, blood calcium, blood urea nitrogen, blood sugar, and white blood cell count versus ulinastatin alone. This interpretation might be attributed to the fact that somatostatin plus ulinastatin in the treatment of patients with severe acute pancreatitis facilitates the recovery of pancreatic function and attenuate the inflammatory response.

The etiology of acute severe pancreatitis in traditional Chinese medicine is mostly believed to be the invasion of exogenous pathogens, overeating, alcoholism, or obstruction of the bile ducts, liver qi stagnation, liver qi reversal, and internal toxins, and evil toxin accumulation, and finally to qi stagnation, blood stasis, and obstruction of qi suffocation in the internal organs. For the syndrome of heat accumulation, Dachengqi decoction is given to clear heat and dehumidify and detoxify the inside. As such, the ecological balance of bacteria in the intestinal tract is maintained, which reduces the occurrence of enterogenic endotoxemia and fights the acute inflammatory reaction, blocks the further development of the disease, reduces complications, and avoids serious trauma caused by surgery. The combination of raw rhubarb with *Bupleurum*, betel nut, *Magnolia officinalis*, *Citrus aurantium*, and other medicines can protect the liver and gallbladder, relax the sphincter of holmium, enhance bile flow, reduce the toxicity of bile acids, and promote the recovery of gastrointestinal digestive function, preventing acute severe illness from severe progression of pancreatitis.

The article "Somatostatin plus Ulinastatin in the Treatment of Severe Acute Pancreatitis and Its Effect on Serum Cytokine Levels" was retracted in 2023. Reasons: unreliable results or conclusions; concerns about the data; concerns about the peer review; concerns about the citations.

Previous studies have shown that inflammatory reactions involved in the occurrence and development of severe pancreatitis [10]. TNF-*α* is mainly secreted by macrophages, and the elevated TNF-*α* can promote the production of inflammatory factors, trigger immune damage, and increase vascular endothelial permeability. Interleukin-6 (IL-6) is mainly secreted by endothelial cells and T cells. At present, IL-6 has been clinically used as one of the important indicators for predicting severe pancreatitis. Elevated IL-6 alters the activity of G proteins, leading to impaired brain cell function and increased incidence of complications such as shock. C-reactive protein (CRP) is an acute phase protein. Under the influence of various factors such as stress state, tissue damage, or infection, the level of serum CRP will increase significantly. In the early stage of severe pancreatitis, the body will release a large number of inflammatory factors, triggering a series of cascade inflammatory reactions, aggravating the primary disease and other organ damage. Therefore, in the treatment of severe pancreatitis, strengthening the detection of inflammatory factors such as CRP, TNF-*α*, and IL-6 is of great significance for evaluating the patient's condition and prognosis. The limitation of this study is that it did not monitor prognostic factors, and future research is required to conduct multivariate analysis of prognostic factors to obtain more clinical data (Table 3)

## 5. Conclusion

Somatostatin plus ulinastatin offers a promising route for treating patients with severe acute pancreatitis. It is worthy of clinical application.

## Figures and Tables

**Table 1:** Comparison of efficacy (*n* (%)).

	Control group (*n* = 50)	Experimental group (*n* = 50)	*x* ^2^	*P*
Cured	20 (40.0)	31 (62.0)		
Effective	19 (38.0)	16 (32.0)		
Ineffective	11 (22.0)	3 (6.0)		
Total effectiveness	39 (78.0)	47 (94.0)	5.316	0.021

**Table 2:** Comparison of IL-10, IL-18, and TNF-*α* (*x* ± *s*).

Groups	*n*	IL-10 (pg/ml)		IL-18 (pg/ml)		TNF-*α* (ng/l)	
		Before	After	Before	After	Before	After
Control group	50	52.34 ± 15.21	104.22 ± 22.37	223.12 ± 38.49	178.72 ± 19.29	75.13 ± 18.94	42.51 ± 12.17
Experimental group	50	52.57 ± 15.19	168.34 ± 20.12	224.10 ± 38.51	101.33 ± 18.60	75.29 ± 18.65	30.28 ± 10.19
*T*		0.076	15.069	0.127	20.422	0.043	5.448
*P*		0.94	＜0.001	0.899	＜0.001	0.966	＜0.001

**Table 3:** Comparison of serum amylase, blood calcium, blood urea nitrogen, blood sugar, and white blood cell count (*x* ± *s*).

Groups	*n*	Serum amylase (pg/ml)		Blood calcium (ng/l)		Blood urea nitrogen (pg/ml)	
		Before	After	Before	After	Before	After
Control group	50	637.88 ± 195.89	487.71 ± 202.12	1.33 ± 0.18	1.50 ± 0.19	28.18 ± 2.43	22.81 ± 3.20
Experimental group	50	639.42 ± 194.83	405.32 ± 177.29	1.35 ± 0.17	1.65 ± 0.22	28.24 ± 2.39	18.02 ± 2.55
*T*		0.039	2.167	0.571	3.649	0.124	8.278
*P*		0.969	0.033	0.569	＜0.001	0.902	＜0.001

Groups	*n*	Blood sugar (pg/ml)			White blood cell count (pg/ml)		
		Before	After		Before	After	

Control group	50	17.80 ± 2.77	15.98 ± 2.32		23.21 ± 2.87	18.75 ± 3.31	
Experimental group	50	17.76 ± 2.61	14.17 ± 1.96		23.29 ± 2.68	15.10 ± 2.55	
*T*		0.074	4.214		−144	6.177	
*P*		0.941	＜0.001		0.886	＜0.001	

The article "Somatostatin plus Ulinastatin in the Treatment of Severe Acute Pancreatitis and Its Effect on Serum Cytokine Levels" was retracted in 2023. Reasons: unreliable results or conclusions; concerns about the data; concerns about the peer review; concerns about the citations.

## Data Availability

No data were used to support this study.
